RETRACTED

# Effect of Basicity on the Microstructure of Sinter and Its Application Based on Deep Learning

**DOI:** 10.1155/2021/1082834

**Published:** 2021-09-09

**Authors:** Jian-Ming Zhi, Jie Li, Jia-Hao Wang, Tian-Yu Jiang, Ze-Yi Hua

**Affiliations:** ^1^School of Metallurgy and Energy, North China University of Science and Technology, Tangshan 063210, China; ^2^College of Science, North China University of Science and Technology, Tangshan 063210, China

## Abstract

The influence of the evolution rule of basicity (0.6∼2.4) on the mineral composition and microstructure of sinter is studied by using a polarizing microscope, and the comprehensive application analysis of the drum index, vertical sintering speed, and yield of sinter shows that, over the course of an increase in basicity (0.6∼1.0), the mineral structure changed from the original porphyritic-granular structure to a porphyritic structure. At the same time, there was no calcium ferrite phase in the bonding phase at a basicity of less than 1.0; therefore, the downward trend of the three indicators is obvious. When the basicity was further increased to approximately 1.6, the main structure of the mineral phase changed from a corrosion structure to an interweaving corrosion structure. Because of the existence of a porphyritic-granular structure, the structure of the mineral phase was extremely inhomogeneous and most complex near the basicity of 1.6; although a small amount of calcium ferrite displayed an acicular structure, the drum index appeared to show a very low value. With an increase in basicity to 2.0, the mineral phase structure was dominated by an interweaving corrosion structure with a uniform framework, and the content of calcium ferrite reached the highest value. Moreover, a clear acicular structure developed, and the drum index also increased to the highest value. At a basicity of more than 2.0, a mineral structure began to appear and the corrosion, porphyritic-granular structure, and the drum index also showed a slightly declining trend. Therefore, in the actual production process, basicity should be avoided as far as possible at around 1.0 and 1.6 and it should be controlled at around 2.0. At the same time, based on the mineral facies data set of this paper, the convolutional neural network is used to carry out a simple prediction model experiment on the basicity corresponding to the mineral facies photos, and the effect is quite good, which provides a new idea and method for the follow-up study of mineral facies.

## 1. Introduction

In the 21st century, with the development of the steel industry and the progress of science and technology, recent research on the composition of sinter minerals and the structure of minerals is also increasing. Among this research, the most common focus is on the influence of basicity and its relationship with metallurgical properties [1–7]. Guo et al. [8] used X-ray diffraction (XRD), an optical microscope (OM), a scanning electron microscope (SEM), and other types of equipment to study the differences in mineral composition and structure of high-basicity (1.84∼2.11) sinters produced by many large domestic steel plants. The results showed that most of the sinters are composed of magnetite, hematite, calcium ferrite, calcium silicate, and glass phases, and as the basicity increases, their morphology changes, displaying xenomorphic crystals. Secondly, the proper addition of Al_2_O_3_ in the liquid phase of the sintering aids in the formation of acerous calcium ferrite. Webster et al. [9] used in situ S-XRD (synchrotron X-ray diffraction) to study the effect of basicity on the crystallization of the effective bonding phase of SFCA (silico-ferrite of calcium and aluminum) and Fe-rich SFCA in the sinter during cooling. The formation of Fe-rich SFCA is inhibited when the basicity is decreased from 4.0 to 2.5, but SFCA crystallizes from the melt during the cooling of material with basicity of 2.5. Liu et al. [10] took the Sijiaying Mine as an example, and the research showed that, with an increase in basicity, the content of calcium ferrite forming the effective binding phase in the sinter increases obviously; then, the strength of the sinter and other metallurgical properties is improved accordingly. All of the above studies focus on the influence of basicity on mineral phase composition and mineralogical structure at a small range. It is not easy to explain the universality of the rule of basicity change in a sinter's mineralogical structure. For the preparation of high-quality sinters, the microstructural analysis represents a safeguard. Therefore, this study on the evolution characteristics of the mineral structure of sinters with a wide range of basicity (0.6∼2.4) focuses on providing an accurate technical reference for production practice.

RETRACTED

At the same time, in order to have a more convenient method to study the mineral facies image in the future, we learned that, in recent years, CNN's accuracy has been tested by large-scale image data sets such as ImageNet [11], which contains more than 100 million images. New CNN such as AlexNet [12], VGg, GoogLeNet [13], and RESNET [14] are used in image classification. We are doing better and better in this respect. And we have achieved good results in face recognition [15], license plate recognition [16], and handwritten character recognition [17]. The recognition rate of the deepID2 + model in the field of face recognition has reached 99.47%, far exceeding the human eye recognition ability [18]. Therefore, at the end of this paper, we use the sample set of phase diagram in this paper to do a simple regression prediction experiment through a convolutional neural network, the purpose is to predict the alkalinity through the mineral photos, the accuracy is about 65%, and the effect is good, so it provides a certain experimental basis for future research in this direction and also provides the corresponding technical guidance for researchers.

## 2. Materials and Methods

The chemical composition and loss on ignition of raw materials for sintering are shown in Table 1.

The main raw materials are Brazil ore fines, local alkali fine powder, and Australian iron ore, which constitute more than 70% and use dolomite powder to adjust the MgO content of the sinter to 2.3% and the carbon content to 3.75%. In the test, the basicity of the sinter (R = w(CaO)/w(SiO_2_)) was adjusted by quicklime to be 0.6∼2.4 and test numbers were recorded as R_0.6_∼R_2.4_. The sintering cup specifications were Φ 200 mm × 600 mm; some of the sintering process parameters for sintering were an ignition negative pressure of 6.0 kPa, an ignition temperature of 1150 ± 50°C, and a sintering negative pressure of 10.0 kPa. In the drum experiment, the device shown in Figure 1 was used for measurement. The specific measurement methods are as follows.

Drum index:

(1) $$\begin{array}{c} T=\frac{m_{1}}{m_{0}}\times 100\%. \end{array}$$

Here, *m*_0_ indicates the drum sample quality, kg, and *m*_1_ indicates that, after turning the drum, the particle size mass was +6.3 mm, kg.

The finished sinter of each sample was cut into rectangles that were slightly larger than 2.5 cm × 1.5 cm × 0.5 cm. First, one side of the glass was coarsely ground and finely ground until it was finely ground on the glass plate, and then it was washed with clean water. The finely polished surface has then adhered to the slide with solid optical gum, which in turn was coarsely ground and finely ground until the thickness was 0.3 mm, and it was then polished in thin sections. Finally, the mineral composition and mineralogical structure were observed and analyzed under a Zeiss axioskop40 polarizing microscope.

## 3. Results and Analysis

The chemical composition analysis (mass fraction) of the finished sinter under different alkalinity in the test is shown in Table 2, and index parameters from the sintering experiments test are shown in Table 3.

### 3.1. Influence of Basicity on Mineral Composition of Sinter

The mineral composition and volume percentage of the sinter are listed in Table 4.

RETRACTED

As seen in Table 4, the mineral composition of sinter formed by different degrees of basicity involved iron oxide phases and binding phases. The main iron oxide phases were magnetite and hematite. The binding phase consisted mostly of calcium ferrite, dicalcium silicate, and smaller amounts of glassy phase. The following conclusions can be made:

1. In the sinter with basicity of 1.0 or less, the main mineral was magnetite, with a small amount of hematite. The binding phase was mainly dicalcium silicate and glassy phase in the silicate liquid phase, without an obvious calcium ferrite phase.
2. In the sinter with basicity of 1.2∼1.6, as the basicity increased, the magnetite generally shows a downward trend, from 75% to 55%. The hematite content is decreasing but fluctuates greatly, and the maximum variation threshold is about 10%. This phenomenon is consistent with the conclusion that basicity increases and skeletal texture Fe_2_O_3_ decreases. Similarly, with the increase in basicity, the Free-CaO in the sintering raw materials increased, which changed the sintering atmosphere to a certain extent. In a weak reducing atmosphere or oxidizing atmosphere, hematite (Fe_2_O_3_) will increase, so the excessive CaO and Fe_2_O_3_ form calcium ferrite. At this point, the presence of calcium ferrite in the binding phase minerals and the significant increase in the content with the increase in basicity also confirm the above statements. Meanwhile, the content of the binding phase, such as dicalcium silicate and glassy phase, decreased obviously, except for a slight increase in dicalcium silicate.
3. In the sinter with basicity of 1.8∼2.4, magnetite content in the iron oxide phases increased, the hematite content was reduced slightly, vitreous quality in the effective binding phase gradually decreased and tended to be minimal, dicalcium silicate and calcium ferrite slightly increased, and the content of calcium ferrite reached a maximum when basicity was 2.0; the content decreased slightly when the basicity was increased, which was related to the microstructure, which was later analyzed in depth.

In conclusion, with the increase in basicity, the mass fraction of magnetite in the iron oxide phases decreased obviously, while hematite increased slightly. The total mass fraction of iron ore decreased from 90% to 65%, due to the increase in basicity, which promoted the formation and stability of calcium ferrite in the effective binding phase. Furthermore, the formation of iron-bearing minerals in the iron oxide phase can be restrained appropriately [19]. Therefore, when the basicity was greater than 1.0, the calcium ferrite phase appeared, its mass fraction increased obviously by around 25%, the content of dicalcium silicate increased slightly, and the content of vitreous substance decreased significantly. When the basicity was 2.0, the calcium ferrite content reached 40∼45%, and it can be seen from Table 2 that the SiO_2_ and CaO content also increased at this time. After the reaction of CaO and SiO_2_ completely, the surplus CaO reacted with Fe_2_O_3_ to form calcium ferrite. Therefore, the content of calcium ferrite increased significantly, which is also in line with the theoretical basis of the ferrite liquid phase as the main binding phase in the high-basicity sinter.

RETRACTED

### 3.2. Evolution Rule of Basicity on the Microstructure

The microstructure under different degrees of basicity was observed and analyzed using a Zeiss axioskop40 polarizing microscope.

For the basicity range of R ≤ 1.0 (0.6∼1.0), according to mineral phase analysis of the sinter samples, the results are shown in Figures 2 and 3.

It can be seen from Figure 2 that the mineral structure was relatively uniform when the basicity ranged from 0.6 to 0.8, displaying mainly porphyritic-granular and porphyritic structures. The crystal shape of magnetite was mainly hypautomorphic and moderately xenomorphic and was distributed uniformly. The crystal size was generally 0.03∼0.08 mm. This was often cemented by glassy phase or glassy phase and dicalcium silicate to form a porphyritic-granular or porphyritic structure. Hematite was not unevenly distributed; rather, it was mostly distributed around the pores, mainly as hypautomorphic crystals on the edge of magnetite to form a reaction rim, with local skeletal crystals, and its crystal size was generally 0.01∼0.03 mm. Within this range of basicity, glassy phase material represented the main bonding phase, and the distribution was relatively uniform.

In combination with the mineral composition listed in Table 3, the data indicate that the magnetite content in the iron oxide phases is significantly greater than hematite, which is clearly visible in the microstructure. The gray-white areas in the mineral phase diagram indicate the magnetite, and the glassy phase plays the role of cementation magnetite in the mineral phase structure and appears in dark gray.

As shown in Figure 3, when the basicity reached 0.9∼1.0, the mineral structure of the sinter changed slightly; in addition to the main porphyritic structure, a local melting corrosion structure also appeared. The mineral structure started to become uneven. The crystal of magnetite was mostly hypidiomorphic, with a crystal size of 0.02∼0.06 mm. It was mostly cemented by a glassy phase and a small amount of dicalcium silicate into a porphyritic structure. The appearance of a local molten corrosion structure indicated that a small amount of magnetite was eroded by calcium ferrite and dicalcium silicate. On the other hand, hematite was mostly xenomorphic and hypautomorphic, with a crystal size of 0.01∼0.03 mm and uneven distribution. It was mostly distributed around the pores, some of which were oriented in a rhombohedral arrangement and a small amount of which was distributed at the edge of magnetite to form a reaction rim. Within this range of basicity, the binding phase contained a glassy phase, dicalcium silicate, and a small amount of melilite. The glassy phase was mainly cemented with magnetite to form a porphyritic structure [20].

RETRACTED

Above all, in sinters with basicity of less than 1.0—meaning that the process of basicity increased from 0.6 to 1.0—the sinter's mineral structure transitioned from porphyritic-granular to porphyritic, and a partial corrosion structure appeared near the basicity of 1.0, from which the mineral structure began to change from single to complex. Because of the corrosion structure, calcium ferrite formation occurred [21], but no obvious calcium ferrite phase was measured in the mineral compositions listed in Table 3. The main reason for this was the formation of trace semicalcium ferrite. No obvious calcium ferrite (CaO·Fe_2_O_3_) crystals were seen in the microstructure of the sinter [22–27]. The discovery of this phenomenon is consistent with the research conclusions of Professor Chen et al. [28] of Central South University on the microstructure of sinter. The main reason for the absence of the formation of calcium ferrite is the fact that the free energy of calcium ferrite is much greater than that of calcium silicate at this alkalinity range, so it is difficult to form calcium ferrite under these conditions; on the contrary, calcium silicate is easily formed and, occasionally, a small amount of semicalcium ferrite liquid appears. Therefore, the appearance of the calcium ferrite phase and local corrosion structure in the mineral composition was also based on this phenomenon.

When the basicity was R > 1.0 (1.2∼1.6), the finished mineral samples were analyzed separately, as shown in Figures 4 and 5.

When basicity ranged from 1.2 to 1.4, the microstructure of the sinter was not uniform. When R = 1.2, the sinter displayed a mainly porphyritic structure with partial corrosion. When R = 1.3, the structure displayed mainly interleaving corrosion with a partially porphyritic structure. When R = 1.4, the structure consisted mainly of corrosion with a partially porphyritic structure. Therefore, it can be seen that the structure of minerals was extremely uneven within this range, due to the coexistence of multiple mineral phase structures. In addition to the mineral composition table, the content of calcium ferrite could be measured obviously when the basicity was 1.2; the accuracy of the data can also be explained by the appearance of the corrosion and interweaving corrosion structures in the microstructure.

RETRACTED

In the iron oxide phases, the crystal shape of magnetite is gradually transformed from idiomorphic and hypautomorphic to xenomorphic, and the idiomorphic and hypautomorphic crystals are cemented into a porphyritic structure by glassy phase and dicalcium silicate, while the xenomorphic crystals are cemented by some glassy phase, calcium ferrite, and a small amount of dicalcium silicate to form a corrosion and interweaving corrosion structure. The change in crystal size was 0.05∼0.1 mm. Hematite formed a local xenomorphic structure when the basicity was 1.3, while the rest showed a hypautomorphic structure. The crystal size of hematite was approximately 0.02 mm, and its distribution was not uniform and mostly distributed around the pores; that is, the magnetite particles around the pores were oxidized into hematite by air, so there was more hematite distributed here, and the hematite was locally connected to sheets. There was no cementation between the magnetite particles, which also provided favorable conditions for the formation of calcium ferrite, and the rest of them were arranged in a diamond orientation.

The binding phase mainly included glassy phase, calcium ferrite, and dicalcium silicate. At basicity of 1.2, the main bonding phase was glassy phase, supplemented by a small amount of calcium ferrite. When the basicity was 1.3 and 1.4, calcium ferrite was the main binding phase, and their shapes changed from fibrous to columnar and platy. The content of calcium ferrite increased obviously, but there were no acicular shapes with better strength.

When the basicity increased to 1.5, the inhomogeneous degree of the mineral phase structure increased, and the interweaving corrosion structure was the main structure, but a large number of corrosion structures could be clearly seen locally. Most of the magnetite was in the form of xenomorphic crystals, which were mainly formed by the interweaving corrosion structure of calcium ferrite, a small amount of dicalcium silicate, and glassy phase. In part, the cementation of vitreous, dicalcium silicate, and calcium ferrite formed a local corrosion structure, and crystalline magnetite, acicular calcium ferrite, and dicalcium silicate were found together in the glassy phase. At this time, the content of hematite declined and its distribution was not uniform; hematite was still mostly distributed around the pores, while some of the hematite was distributed in strip form in magnetite. Calcium ferrite, as the main binding phase, was locally acicular and concentrated with dicalcium silicate. Dicalcium silicate mainly took the form of xenomorphic crystals, with coarse crystal size and uneven distribution, mostly with granular and acicular shapes.

RETRACTED

In the entire basicity range, the degree of inhomogeneity of the sinter phase structure reached the maximum at basicity of 1.6, mainly with an interweaving corrosion structure, and local granular and porphyritic structures could be seen; there were many cracks in the ore block. Most of the magnetite was xenomorphic and some was hypautomorphic, which formed a porphyritic or granular structure with the binding phase. Hematite took the form of mainly xenomorphic and hypautomorphic crystals, and the distribution was not uniform, mostly concentrated around the pores. Local hematite was arranged in a rhombohedral orientation, and a small amount of hematite was distributed in a strip in a glassy phase. Compared with the sinter with basicity of 1.5, the change in calcium ferrite content was not obvious, but a small amount of acicular appeared. The content of the vitreous phase increased and was concentrated in magnetite, which resulted in the appearance of a porphyritic and granular structure.

In addition to the above analysis, when the basicity increased from 1.0 to 1.6, the following observations were made [29].

According to the change in the content of calcium ferrite, a small amount of calcium ferrite appeared from basicity of 1.2. With the increase in basicity, calcium ferrite appeared as the main binding phase from 1.3 to 1.6, and the content of calcium ferrite increased obviously at 1.4. However, the best acicular calcium ferrite was not found; instead, it transitioned from a plate column structure to a small number of acicular structures when the basicity was 1.6, accompanied by a small number of acicular transitions from the columnar plate structure at an alkalinity of 1.6. Furthermore, under basicity conditions, the structure of the mineral phase was varied, which led to a decrease in the uniformity of the entire structure and a decrease in the overall performance of the sinter.

In the iron oxide phases, magnetite, as the main mineral, formed the main part of the microstructure of the sinter with the minerals of the binding phase and, compared with the content of magnetite in the sinter when the basicity is less than 1.0, the content of magnetite gradually decreased with the increase in basicity. Thus, the basicity is indeed one of the factors by which to improve the sintering reaction while it is being carried out, and it accounts for a high proportion of this improvement. The idiomorphic and hypautomorphic crystals were the basis of the transition to hypautomorphic crystals in the change in the magnetite crystal. The fact that the magnetite was dominated by hypautomorphic crystals at basicity of 1.5 indicates that the trend of the change in the crystal form is also based on this. For hematite, the relationship between the content of hematite and the sintering reaction was positive and its content decreased when the reaction was sufficient and increased when the reaction slowed down. The reasons for this are as follows: (1) the formation of calcium ferrite is the result of the reaction between CaO and Fe_2_O_3_, so the hematite decreases when the content of calcium ferrite increases, and vice versa; (2) the distribution of hematite around the pores in the microstructure promotes the development of secondary hematite to a certain extent, thus increasing the content of hematite.

RETRACTED

When the basicity R > 1.8 (1.8∼2.4), the finished mineral samples were analyzed, respectively, as shown in Figures 6 and 7.

When the basicity was 1.8, the mineral structure was more homogeneous than before, and most samples showed an interweaving corrosion structure. Only a small number of localized corrosion structures were better than the porphyritic and granular structures. Most of the magnetite was in the form of xenomorphic crystals with fine crystal size, ranging from 0.01 to 0.05 mm. Most magnetite was cemented by calcium ferrite and dicalcium silicate to form an interweaving corrosion structure. The crystal structure of hematite was also xenomorphic-hypautomorphic, the crystal size was generally 0.02∼0.22 mm, the distribution was not uniform, mostly distributed around the pores, and the xenomorphic hematite was connected locally. Compared with the basicity of 1.6, the content of calcium ferrite was obviously increased and it was the main binding phase, which mostly can be seen as obvious xenomorphic crystals and local acicular structures.

The mineral structure of the sinter with basicity of 2.0 was more stable, mainly with an interweaving corrosion structure. The magnetite was mainly xenomorphic and somewhat hypautomorphic. The crystalline grain size was generally 0.03∼0.06 mm, and the interweaving corrosion structure was formed by the cementation of calcium ferrite and dicalcium silicate. The hematite content was low, the crystal size was generally 0.01∼0.03 mm, and most of the hematite crystals were distributed around the pores. At this time, the content of calcium ferrite reached the highest value of approximately 45% in the entire basicity range. The appearance of a large area of calcium ferrite in the microstructure also proved the accuracy of these data; a large amount of acicular calcium ferrite was found in the structure, with a small number of strip shapes, and the crystal shape started to become thick and dense.

RETRACTED

Continuing to increase the basicity, as shown in Figure 7, when the basicity reached 2.2∼2.4, the highest range of basicity, the mineral structure became nonuniform when compared with basicity of 2.0. Although the main body still displayed an interweaving corrosion structure, local corrosion and a porphyritic-granular structure began to appear; in addition to basicity of 2.4, a small number of cracks could be seen.

In the iron oxide phases, magnetite underwent a transition from xenomorphic to hypautomorphic and idiomorphic, and the crystal shape started to deteriorate. However, most of the magnetite was cemented with calcium ferrite and dicalcium silicate to form an interweaving corrosion structure, while a few of them began to bind with glassy phase and dicalcium silicate to form a porphyritic-granular structure. However, hematite mostly displayed a combination of xenomorphic and hypautomorphic crystals, the crystal size was still fine, the distribution remained uneven, mostly concentrated around the pores and, in the micrograph of the microscopic phase diagram, hematite was obviously concentrated, and the content was also reduced. Calcium ferrite was still the main composition in the binding phase, but compared with 2.0, its content decreased to 30∼35%, reaching the average level at a better sintering reaction time, and its morphology changed from acicular to strip and columnar. Second, it was evident that the vitreous was reduced at this range of basicity, while the amount of dicalcium silicate increased. It could also be observed that when the basicity was higher than 2.0, the degree of sintering reaction began to decrease. The reduction in hematite content led directly to a reduction in calcium ferrite content, which indicated that the Fe_2_O_3_ involved in the reaction was reduced and the amount of calcium ferrite produced was also reduced. Due to the insufficient sintering reaction, excessive CaO was generated under high basicity, and CaO could stabilize *β*-2CaO·SiO_2_, leading to an increase in the content of calcium silicate (mainly *β*-2CaO·SiO_2_ and 3CaO·SiO_2_). In addition, because *β*-2CaO·SiO_2_ does not pulverize during cooling, it has good strength [30], which provides some theoretical support for the development of high-basicity sinters.

According to the microscopic analysis of the high-basicity sinter, during the course of increasing basicity from 1.8 to 2.4, the following observations could be made:

1. The degree of homogeneity of the entire mineral phase structure is much higher than that of sinters with basicity from 0.6 to 1.6, which are dominated by an interweaving corrosion structure formed by the mutual development or interweaving of magnetite and binding phase mineral crystals; among them, the mineral structure is the most uniform at basicity of 2.0, and the parameters are excellent. The content of calcium ferrite reaches the maximum at this point, and the mineral content of other bonding phases, such as glassy phase, is the lowest, and it is seldom observed in the microstructure, which is the main reason for the strong performance of the sinter at basicity of 2.0.
2. In the microstructure of the sinter, when the basicity is more than 2.0, the mineral phase structure changes from single to complex. In addition to the best interweaving corrosion structure in the main part, a slight corrosion structure and porphyritic-granular structure begin to appear, and the uniformity of the overall structure shows a downward trend; however, calcium ferrite is still the primary high-quality mineral in the cohesive phase, which is an important reason to promote the development of high-basicity sinters.
3. According to the synthesis of the mineral composition and microstructure, the proportion of dicalcium silicate in the high-basicity sinter increases with the increase in calcium ferrite content, which is due to the increase in basicity and the increase in CaO activity. Moreover, the formation of dicalcium ferrite at a high melting point is increased, so the stability of calcium ferrite is improved, and the two complement each other and increase at the same time.

RETRACTED

### 3.3. Analysis of the Variation Law of Drum Strength

According to the drum index of a sinter under different basicity conditions, the trend of drum index can be visualized as shown in Figure 8.

As shown in Figure 8, in the entire basicity range of 0.6∼2.4, the drum index of the sinter remains stable at 0.6, while it continues to increase, presenting two decreasing areas—0.8∼1.0 and 1.5∼1.8—after 2.0, and there is a stable trend at the higher level. Based on the analysis of the above-mentioned evolution rules of minerals, the following conclusions can be made.

When the basicity is 0.6, the sinter phase structure is single and uniform, mainly a porphyritic-granular structure. The mineral content of the bonding phase is less, and the iron oxide phases content increases; therefore, the sinter drum index remains stable at this time.

At basicity in the range of 0.8∼1.0, the mineral phase structure of the sinter is mainly porphyritic and granular, with poor strength, and at 1.0, a partial corrosion structure appears, and the mineral phase structure is varied and uneven. Within this range, with the increase in basicity, the content of magnetite in the iron oxide phases of the sinter mineral composition decreases, while the content of hematite increases, the content of glassy phase in the bonding phase increases obviously, and the calcium ferrite phase does not appear; therefore, the drum index in this area presents a low concave area.

RETRACTED

At basicity in the range of 1.4∼1.6, with the increase in basicity, the content of iron oxide phase hematite in the mineral composition of the sinter increased and the content of the bonding phase decreased. In particular, the content of calcium ferrite in the effective bonding phase decreases obviously when basicity is 1.6, the mineral composition is complex, and the mineral phase structure is transformed from the main corrosion structure. The local porphyritic structure gradually transforms into the main interweaving corrosion structure and local corrosion structure. When the basicity is near 1.6, the sinter phase structure mainly takes the form of interweaving corrosion, with a partially porphyritic structure and local granular structure, and the mineral phase structure is extremely inhomogeneous and complex. This is the main reason for the additional low concave area when basicity is around 1.6.

When the basicity reaches 2.0, the interweaving corrosion structure dominates the mineral phase structure, the content of calcium ferrite in the bonding phase reaches the highest value, and the basicity continues to increase. The mineral phase begins to demonstrate a porphyritic structure, corrosion structure, and porphyritic-granular structure, and its structure begins to become complex; the calcium ferrite content also begins to decrease. Therefore, the sinter with basicity of 2.0 demonstrates the best range of performance indexes in the entire basicity range due to the homogeneous mineral phase structure and the highest content of calcium ferrite.

### 3.4. Analysis of Vertical Sintering Speed and Yield

According to the vertical sintering speed and yield rate of sinter under each basicity condition, the comparative analysis graphs were drawn as shown in Figure 9.

As shown in Figure 9, in the entire basicity range from 0.6 to 2.4, the vertical sintering speed accelerates and the sinter yield rate improved with increasing basicity, and this evolution rule was consistent with the pattern obtained from the above changes between basicity and drum index, which showed a small difference; that is, before the basicity of 1.6, the sintering phase structure was complex and the effective binding phase was less, so it leads to a slow vertical sintering speed and a decrease in yield, while after reaching 2.0, the vertical sintering speed and yield showed better index parameters. So overall the main variation trend was the same without difference.

RETRACTED

Then, after the basicity was increased, the quicklime content in the mixture increased, which strengthened the granulation effect and improved the permeability of the material layer, which lead to the improvement of the vertical sintering speed, and according to the structure of the mineral phase at this time, the interweaving corrosion structure was the main structure, and the effective binding phase was mainly the calcium ferrite phase, so the role of the liquid phase condensation of the sinter was maximized at this time, and therefore the yield rate increases. Therefore, through the study of vertical sintering speed and yield rate, it was also obtained that basicity 2.0 was the optimal basicity condition to complete the performance indexes of the sinter.

## 4. Experiment of the Basicity Prediction Model

### 4.1. Convolutional Neural Network Model

Neural network is an algorithm that imitates the human brain nervous system, including input unit, hidden unit, and output unit [31–34]. It imitates a way of transmitting and processing information between neurons in the brain nervous system. Each cell contains a large number of nodes, there is a weight between nodes, and each node has an incentive function. The operation mode is shown in Figure 10.

Convolutional neural networks (CNNs) are artificial neural networks with forward structure. Generally, CNN is divided into input layer, middle layer, and output layer. Generally, the input layer is used to receive images and is composed of convolution layer. The middle layer includes convolution layer, full connection layer, and pooling layer. The convolution layer is used to extract the features of the image, the full connection layer is used to receive all the features, and the pooling layer is used to compress the features of the image, which can save the main features and reduce the complexity of network computing. The output layer is generally composed of full join layer, which is used to generate a classifier to classify the output value.

In this experiment, the VGG16 model structure is used to extract the features of mineral facies photos, and the basicity value of image regression is given with the extracted features. The training process is shown in Figure 11.

From left to right, a color picture is input to the network, the white box is the convolutional layer, the red is the pooling, the blue is the fully connected layer, and the brown box is the prediction layer. The function of the prediction layer is to convert the information output by the fully connected layer into corresponding category probabilities. The loss function used should be the mean square error (mse). The optimization method uses the Adam algorithm to achieve the role of regression prediction.

RETRACTED

### 4.2. Experimental Data

The data set used in this experiment is derived from the above-mentioned mineral facies photos at each basicity in this article. In addition to the data set in the article, there are all the photos in the experiment, a total of 659 photos, and the picture format is jpg format.

Because the unbalanced data will lead to overfitting or underfitting phenomenon in the process of network training, in order to get better effect of mineral facies photos, we use rotation, translation angle, change direction, and other operations to increase the number of intact photos to 800, which effectively solves the problem of poor experimental performance caused by unbalanced data. In addition, the size of each image is converted to 224 × 224, and all are normalized.

### 4.3. Experimental Process and Results

Firstly, the folder of different basicity is established, and then the photos of ore facies with good basicity are put in. After the training of the VGG16 model, the predicted accuracy and loss rate are finally output. The specific training process is shown in Figure 12.

For the VGG16 model, the more the number of training samples and the more balanced the data set, the higher the test accuracy. In order to fully train the images and test the accuracy of the images, 70% of the original mineral phase diagram in each basicity folder was used as the training set to train the VGG16 model and 30% as the verification set. Finally, after thousands of iterations, the prediction results are shown in Figures 13 and 14. The prediction accuracy of the image can reach about 65%, and the loss value is about 1.4.

On the whole, through the above experiments, we can get the convolutional neural network regression algorithm experiment which has obvious outstanding effect in the research direction of mineral image basicity prediction, so it provides a new idea and method for the future research of mineral image processing.

## 5. Conclusions

Through the study and analysis of mineral composition and the evolution rule of the microstructures of sinters under different basicity conditions, the following conclusions can be drawn:

1. Granular and porphyritic mineral structure is dominant when basicity varies from 0.6 to 1.0. In this study, the basicity changed from a porphyritic-granular to a molten corrosion structure at the range of 1.2∼1.6; among them, the interweaving corrosion structure appeared at basicity of 1.4, but it still coexisted with the corrosion structure and the porphyritic-granular structure. When the basicity continued to increase to 2.0, the main body presented the best interweaving corrosion structure, and the distribution was uniform. When the basicity exceeded 2.0, although the main body was still dominated by an interlaced corrosion structure, local corrosion and a porphyritic-granular structure began to appear.
2. The rule of variation in mineral crystal morphology with basicity is that, under low-basicity conditions, the iron-bearing minerals present idiomorphic and xenomorphic crystals and begin to transform into xenomorphic crystals at high basicity. The calcium ferrite in the binding phase appeared as semicalcium ferrite when the basicity was 0.6∼1.0. However, calcium ferrate began to appear at basicity of 1.2, but its morphology was mainly plate-columnar-shaped when we continued to increase the basicity to 1.6 around the beginning of the local acicular phase. When the basicity reached 2.0, a large amount of acicular calcium ferrite appeared, and strip and columnar formations began to appear locally. The continued increase in basicity was mainly manifested in strip and columnar formations.
3. After the secondary study of sinter drum index, yield rate, and vertical sintering speed, the same revolution rule was obtained that with the change of basicity, sinter strength showed double low concave area; that is, when basicity in the range of 0.8∼1.0 and 1.4∼1.6 where the sinter phase structure does not perform well, production under this condition should be avoided as much as possible. And basic was around 2.0, where the overall performance of mineral phase structure was good, which was the best indicator for sinter to achieve double excellent mineral phase structure and strength.
4. The convolutional neural network based on the vgg16 model can predict the basicity of ore phase image. The accuracy of prediction can reach about 65%. Because of the small sample set, the prediction accuracy is not very high. However, through this experiment, it can be determined that the VGG16 model can deal with the problems similar to this mineral phase diagram, and the prediction results are of referential value. It laid an important foundation for the follow-up research.

RETRACTED

## Figures and Tables

**Figure 1:** Equipment diagram of drum experiment.

**Figure 2:** R_0.6∼0.8_ sinter microstructure (reflected light × 100). (a) R_0.6_ porphyritic-granular structure; (b) R_0.6_ local porphyritic structure; (c) R_0.6_ porphyritic structure; (d) R_0.8_ local porphyritic structure; (e) R_0.8_ hematite distributed on the edge of magnetite.

**Figure 3:** R_0.9_∼R_1.0_ sinter microstructure (reflected light × 100). (a) R_0.9_ porphyritic structure; (b) R_0.9_ hematite distributed on the edge of magnetite (reflected light × 200); (c) R_1.0_ porphyritic structure; (d) R_1.0_ local porphyritic structure; (e) R_1.0_ local corrosion structure.

**Figure 4:** R_1.2∼1.4_ sinter microstructure (reflected light × 100). (a) R_1.2_ porphyritic structure; (b) R_1.2_ corrosion structure; (c) R_1.2_ centralized distribution of calcium ferrite; (d) R_1.3_ interweaving corrosion structure; (e) R_1.3_ porphyritic structure; (f) R_1.4_ corrosion structure; (g) R_1.4_ porphyritic structure (reflected light × 50).

**Figure 5:** R_1.5∼1.6_ sinter microstructure (reflected light × 100). (a) R_1.5_ interweaving corrosion structure; (b) R_1.5_ corrosion structure; (c) R_1.5_ centralized distribution of acicular calcium ferrite; (d) R_1.6_ interweaving corrosion structure; (e) R_1.6_ local granular structure; (f) R_1.6_ hematite with rhombohedral orientation.

**Figure 6:** R_1.8∼2.0_ sinter microstructure (reflected light × 100). (a) R_1.8_ interweaving corrosion structure; (b) R_1.8_ local corrosion structure; (c) R_2.0_ interweaving corrosion structure; (d) R_2.0_ centralized distribution of calcium ferrite.

**Figure 7:** R_2.2∼2.4_ sinter microstructure (reflected light × 100). (a) R_2.2_ interweaving corrosion structure; (b) R_2.2_ corrosion structure; (c) R_2.2_ centralized distribution of hematite; (d) R_2.4_ interweaving corrosion structure; (e) R_2.4_ local granular-porphyritic structure; (f) R_2.4_ centralized distribution of hematite.

**Figure 8:** Relationship between basicity and sinter drum index.

**Figure 9:** Relationship between basicity and vertical sintering speed and yield.

**Figure 10:** Operation mode of the neural network structure.

**Figure 11:** VGG16 model structure.

**Figure 12:** Model training process.

**Figure 13:** Prediction accuracy.

**Figure 14:** Predicted loss value.

**Table 1:** Chemical composition (%) and burning loss of raw materials for sintering.

Material	TFe	SiO_2_	Al_2_O_3_	CaO	MgO	TiO_2_	LOI
Brazil ore fines	62.92	5.65	1.54	0.45	0.11	0.08	0.48
Local alkali fine powder	63.96	3.25	0.79	2.69	1.83	0.09	−0.00
Other fine powders	63.54	5.41	0.75	0.60	2.61	0.34	−0.02
Australian iron ore	57.49	5.04	2.60	0.45	0.11	0.17	9.57
Return ore	54.54	5.53	1.98	11.22	2.15	0.18	−0.01
Sintering dust	42.50	5.94	2.32	18.02	4.24	0.20	5.04
Under the gray	40.92	8.96	2.48	6.96	2.20	0.27	15.70
Miscellaneous ash	—	4.22	0.77	73.30	2.90	0.04	18.31
Dolomite	—	2.68	0.82	38.45	20.21	0.04	35.39
White gray	—	4.22	0.77	73.30	2.90	0.04	18.31

RETRACTED

**Table 2:** Main chemical composition (mass fraction) of sinter (%).

Experiment number	TFe	SiO_2_	Al_2_O_3_	CaO	MgO	TiO_2_
R_0.6_	62.97	5.65	1.93	3.39	1.45	0.16
R_0.8_	61.84	5.64	1.92	4.51	1.87	0.15
R_0.9_	61.24	5.63	1.92	5.07	2.13	0.15
R_1.0_	60.72	5.62	1.91	5.62	2.30	0.15
R_1.2_	59.93	5.61	1.90	6.73	2.30	0.15
R_1.3_	59.62	5.57	1.87	7.25	2.30	0.15
R_1.4_	59.19	5.58	1.87	7.82	2.30	0.15
R_1.5_	58.85	5.56	1.85	8.34	2.30	0.15
R_1.6_	58.39	5.58	1.86	8.93	2.30	0.15
R_1.8_	57.39	5.60	1.87	10.08	2.30	0.15
R_2.0_	56.72	5.56	1.83	11.11	2.30	0.15
R_2.2_	56.03	5.56	1.82	12.23	2.30	0.15
R_2.4_	55.26	5.56	1.81	13.34	2.30	0.14

**Table 3:** Index parameters of sinter.

Basicity	0.6	0.8	0.9	1.0	1.2	1.3	1.4	1.5	1.6	1.8	2.0	2.2	2.4
Drum index/%	61.4	56.8	56.7	56.3	57.0	58.5	56.7	53.8	54.0	55.4	61.2	61.4	64.0
Vertical sintering speed/mm·min^−1^	19.7	20.3	18.3	20.1	19	18.8	20.2	21.5	22.6	27.1	25.7	25.7	27.8
Yield/%	83.7	84.2	80	79.3	78.1	81.1	80.5	80.7	81.3	82.5	84.3	85.2	84.8

**Table 4:** Mineral composition and percentage by volume.

Experiment number	Iron oxide phases		Binding phase					
	Magnetite	Hematite	Calcium ferrite	Dicalcium silicate	Glassy phase	Melilite	CMS	Free-CaO
R_0.6_	80–85	3–5	—	5–7	7–10	—	—	—
R_0.8_	80–85	5–10	—	2-3	5–7	—	—	Bit
R_0.9_	80–85	5–7	—	1-2	10–12	—	—	—
R_1.0_	75–80	8–10	—	1-2	10–12	1-2	—	—
R_1.2_	75–80	2-3	5–10	3–5	8–10	Bit	—	—
R_1.3_	55–60	15–20	10–15	7–10	2-3	1.2	—	—
R_1.4_	50–55	2–5	30–35	5–8	3–5	—	—	—
R_1.5_	55–60	2-3	30–35	7–10	2-3	—	—	—
R_1.6_	55–60	12–15	15–20	5–7	3–5	—	—	—
R_1.8_	35–40	10–12	30–35	15–20	2-3	—	Trace	—
R_2.0_	45–50	Bit	40–45	10–12	Bit	—	—	—
R_2.2_	45–50	2–4	30–35	15–20	1-2	—	—	—
R_2.4_	50–55	5–10	30–35	10–12	Bit	—	bit	—

CMS is monticellite.

## Data Availability

The mineral image data used to support the findings of this study have not been made available because these data in this paper are obtained through experiments, without the use of external data for research.
